The article "Government Structure, Political Connection, and Enterprise Resource Acquisition of Multidimensional Environmental Impact: An Empirical Study Based on the Structural Equation Model" was published in 2022. Journal: J Environ Public Health.

# Government Structure, Political Connection, and Enterprise Resource Acquisition of Multidimensional Environmental Impact: An Empirical Study Based on the Structural Equation Model

**DOI:** 10.1155/2022/4471412

**Published:** 2022-07-07

**Authors:** Qiuying Lv, Chen Chen

**Affiliations:** ^1^School of Social and Public Management, East China University of Science and Technology, Shanghai 200237, China; ^2^Business School, Fuyang Normal University, Fuyang 236000, China

## Abstract

Preferential access to scarce resources can bring competitive advantages and better performance to enterprises. However, the existing literature has a relatively single research path on the influencing factors of enterprise resource access, which has lack of sufficient research from the perspective of multidimensional environment. In particular, as an important factor affecting enterprises' access to external resources, few studies have given empirical results on the impact of political factors such as government structure on enterprise resource access. Preferential access to scarce resources can bring competitive advantages and better performance to enterprises. However, the existing literature has a relatively single research path on the influencing factors of enterprise resource access, which lacks sufficient research from the perspective of multidimensional environment. In particular, as an important factor affecting enterprises' access to external resources, few studies have given empirical results on the impact of political factors such as government structure on enterprise resource access. Through the discussion of multidimensional environmental factors, this paper can provide theoretical reference for the reform of government institutions and the establishment of good political relations between enterprises and the government. Focusing on the multidimensional environment of government structure, political relations, and enterprise resource acquisition, this paper takes 129 enterprises in Central China as samples and uses the structural equation model to empirically verify the relationship between the formalization of government structure, liaison mechanism, decentralization, and enterprise resource acquisition, especially the easing effect of political relations. The results show that the formalization of government structure is promoting enterprises to obtain policy resources and financial resources; the liaison mechanism helps enterprises to obtain financial resources and market resources; decentralization has a significant positive impact on enterprises' access to policy resources and market resources; and political connection magnifies the positive effect of government structure on enterprise resource acquisition, but there are differences in different dimensions.

The article "Government Structure, Political Connection, and Enterprise Resource Acquisition of Multidimensional Environmental Impact: An Empirical Study Based on the Structural Equation Model" was published in 2022. Journal: J Environ Public Health.

## 1. Introduction

Based on the resource theory, preferential access to valuable resources can bring competitive advantage to enterprises and can be translated into better performance [1], so the influencing factors of enterprise resource access have been a hot topic of academic research. Scholars mainly study the external resource acquisition of Chinese enterprises from two aspects: first, the factors of the enterprise itself, such as the internal resources of the enterprise and managers' relations and talents; second, the influence of nonmarket environmental factors, such as collaborative innovation network and social capital, on key resources and information of enterprises. The government-enterprise network, political ties, and government policies affect the enterprise's resource acquisition [2, 3]. Among them, scholars pay special attention to the political factors in the nonmarket environment. Almost every enterprise is influenced by government policy and regulation [4], ignoring the relationship with the government may have a negative effect on the competitive advantage of enterprises. Government networks and political connections are the relational assets of political factors, and enterprises can decide whether to construct the relational networks or take political actions to obtain the resources. However, the author found in the investigation that the government structure, which cannot be controlled by the enterprise, is also affecting the acquisition of enterprise resources. Studies have shown that government is not a single entity and that the relationships between government agencies affect their ability to provide benefits to business [5]. These studies have improved our understanding of the effects of government structural factors on firm resource acquisition, but we still know little about what other structural factors affect firm resource acquisition and the magnitude of the effects.

The purpose of this paper is to break through the limitations of the research on the influence of political factors, focus on multidimensional environmental factors, regard the government structure as a variable, and use political connection factors to explore the relationship between it and government structure and enterprise resource acquisition. On the basis of literature analysis, interviews, and expert opinions, this paper puts forward three factors (formalization, liaison mechanism, and decentralization) of government structure influencing enterprise resources and uses the theory of political connection to deepen the understanding of the relationship between them. We tested our hypothesis through a questionnaire survey of 129 enterprises in central China, in order to fill in the gap in the research on the relationship between government structure and enterprise resources and to gain a deep understanding of the law of government structure change. It is also helpful for enterprises to understand the operating mode and characteristics of government structure and to take targeted strategies to establish political ties and access to resources.

The article "Government Structure, Political Connection, and Enterprise Resource Acquisition of Multidimensional Environmental Impact: An Empirical Study Based on the Structural Equation Model" was published in 2022. Journal: J Environ Public Health.

The rest of this article is organized as follows. Section 2 provides theoretical motivations and research assumptions, followed by an overview of the research design, data collection, and data analysis and followed by a substantive interpretation of the data and discussion of the findings.

## 2. Theoretical Background

### 2.1. Dimensions of Government Structure

The early administrative theory pointed out that the formal organizational structure has the basic characteristics of hierarchy, specialization, and formalization [6], which is the basic starting point of the evolution of organizational theory. Organization hierarchization requires each individual to have a clear position in the pyramid-shaped relationship control structure, which is a kind of hierarchical structure based on authority difference and has the principle of unified command. Specialization involves how the various positions are organized into work units and departments and where jobs with the same attributes or relationships should be located within the same department [7]. A hierarchical and professional organization must meet some formal specifications to ensure consistent results. In addition to the vertical control of the hierarchical and horizontal relationship to coordinate the functional departments, there exist the power differences caused by the rank and function within the organization.

In the study of organizational structure effectiveness, more scholars choose to use case study and questionnaire survey methods. Among them, there are 12 dimensions of organizational structure discussed by the scale method, such as formalization, specialization, standardization, personnel ratio, decentralization, complexity, authorization, and vertical range, which can be summarized and merged into four measurement dimensions, such as complexity, formalization, decentralization, and liaison mechanism [8–11].

Since the introduction of the reform and opening-up policy, the Chinese government has carried out eight organizational reforms, mainly to solve the problems of overstaffed institutions, numerous departments, overlapping responsibilities, and unclear functions. The Chinese government improves government performance by streamlining institutions and personnel, transforming government functions, and rationalizing departmental responsibilities. At present, China's government level is generally a five-level system of the central, provincial, municipal, county, and township levels, but in fact, the government level has the characteristics of the same level of heterogeneity, the combination of virtual reality, the coexistence of rank, and dislocation. The Chinese government has formally completed the institutional reform of merger and reorganization, but has not made any real changes in terms of structural adjustment and decentralization.

The article "Government Structure, Political Connection, and Enterprise Resource Acquisition of Multidimensional Environmental Impact: An Empirical Study Based on the Structural Equation Model" was published in 2022. Journal: J Environ Public Health.

This paper selects and adjusts the measurement dimensions through the content of previous interviews and puts forward three dimensions of enterprise resource acquisition, which are formalization, liaison mechanism, and decentralization, by means of organizational structure theory research, combined with the reality of the Chinese government, and on the basis of listening to experts' opinions. What needs to be explained here is that we define the government structure as the local governments at the municipal (district) and county levels below the provincial level because the government agencies in this area have more contacts with enterprises in urban economic management so that certain dimensions can be verified.

### 2.2. Enterprise Resources

This paper studies the impact of government structure on resource acquisition, so we use the results of corporate political behavior to determine the types of corporate resources. Generally speaking, the results of corporate political behavior are divided into three categories: policy performance, financial performance, and market performance [12]. Accordingly, we define the types of enterprise resources in this paper as: policy resources, financial resources, and market resources. Among them, policy resources are government subsidies, tax exemptions, bailouts or support [13–15], lower administrative and regulatory barriers [16], and changes in public policy to help firms maintain their competitive advantage [17]. Financial resources refer to the availability or low cost of long-term debt financing [18–20]. Market resources refer to the resources obtained by an enterprise that have an impact on market competition, business promotion, and sales. Examples include greater pricing power [16], participation in international competition and trade expansion [21], and income from obtaining business licenses or government contracts [17].

### 2.3. Political Connection

Because governments control critical information and resources, it is difficult for companies to gain a sustainable competitive advantage if they do not pay attention to the political process and dynamics in the operating environment and adopt political strategies. Therefore, the act of political linkage is crucial for companies to gain access to key resources and facilitate economic exchanges [22]. The idea of a positive relationship between political connection and firm performance has been demonstrated [12, 17], which provides firms with various forms of institutional support and valuable resources and information. In the study of the relationship between government structure and enterprise resource acquisition, this paper takes political relations as moderating variables and analyzes the relationship between variables.

The article "Government Structure, Political Connection, and Enterprise Resource Acquisition of Multidimensional Environmental Impact: An Empirical Study Based on the Structural Equation Model" was published in 2022. Journal: J Environ Public Health.

## 3. Research Assumptions

### 3.1. Formalization

Formalization refers to the degree of formalization in the organizational structure, including clear working procedures and instructions, various rules and regulations, working rules, guidelines. The degree of formalization is usually measured by the degree to which regulations are written and the way by which quality and performance are monitored. Therefore, the clearer the workflow of government agencies and the higher the degree of specialization of staff, the higher the efficiency of government work. For example, many enterprises pay special attention to the government's discount loan policy because the interest is very low and there is no repayment pressure, which is very suitable for the business turnover of enterprises. However, the discount loan policy has many conditions and restrictions. If the relevant government departments do not give a detailed explanation of the latest policy, it will increase the various costs for enterprises to apply for discount loans. Similarly, in the process of applying for discount loans, the simplification of government procedures and the degree of specialization of staff will directly or indirectly affect the probability of successful application. At the same time, formalization can effectively reduce the impact of individual differences on the organization. A high degree of formalization means that individuals in an organization have low autonomy in the content and means of work. On the contrary, it means that individuals have greater authority in handling organizational affairs. For example, when an enterprise applies for government project funding, if the government agencies carry out procedures such as document release, selection, and publicity according to uniform requirements and standards, then the enterprise does not need to contact the person in charge of the agency deliberately, and the absence of such informal contact does not hinder the enterprise from applying for the project. Based on the above discussion, the following assumptions are put forward:

  H1: the formalization of government structure has a positive influence on promoting the acquisition of enterprise policy resources
  H2: the formalization of government structure has a positive influence on promoting the acquisition of financial resources of enterprises
  H3: the formalization of government structure has a positive influence on promoting enterprises' access to market resources

The article "Government Structure, Political Connection, and Enterprise Resource Acquisition of Multidimensional Environmental Impact: An Empirical Study Based on the Structural Equation Model" was published in 2022. Journal: J Environ Public Health.

### 3.2. Liaison Mechanism

The liaison mechanism mainly refers to the communication and liaison mechanism among the various departments in the organization. As a result of the horizontal division of labour brought about by specialization, different functional units have been created within the organization that are independent of each other, and the organizational structure needs to coordinate these different functional units so that they are less conflict-ridden and interdependent. The degree of interdependence among the various branches of government may be determined by their degree of differentiation. Some scholars have suggested that the government governance model is between the administrative and the market boundary. The department presents the different system logic and the behavior result: first is to administer according to institutionalized procedures, which is based on the administrative mechanism of bureaucracy; second is to administer in a market-based manner, which is the management mechanism extended by breaking the fetters of bureaucracy. The departmental mechanism of bureaucratic logic is considered to be traditional and procedural, and departments act in accordance with procedures and responsibilities. The latter kind of management mechanism is unconventional and flexible, and departments have similar functions and communicate closely with enterprises under this kind of market logic. Two different departmental operating mechanisms bring different values, rules, and institutional arrangements, which increase the difficulty of coordination. For example, if a business wants to promote a new business related to local economic planning through the government, the government department in charge of the business tends to support the business, while the department with approval authority has bureaucratic logic due to functional differences. Applications for this business may be rejected by examination and approval department, if the necessary liaison mechanisms between departments are not in place. Similarly, in the process of government discount or interest-free loans, the provision of materials, interpretation of policies, and specific handling involve different levels and different machines. If the standards are not uniform and there are barriers to communication, the cost of business handling will increase. Based on the above discussion, the following assumptions are put forward:

  H4: the liaison mechanism of government structure has a positive influence on promoting the acquisition of enterprise policy resources
  H5: the liaison mechanism of government structure has a positive influence on promoting the acquisition of enterprise financial resources
  H6: the liaison mechanism of government structure plays a positive influence on promoting enterprises' access to market resources

The article "Government Structure, Political Connection, and Enterprise Resource Acquisition of Multidimensional Environmental Impact: An Empirical Study Based on the Structural Equation Model" was published in 2022. Journal: J Environ Public Health.

### 3.3. Decentralization

Generally speaking, the control system at the organizational level can ensure the rapid execution of orders from top to bottom. However, in the complex and diverse unitary centralized system, it is a big problem in the practice of state governance to deal with the contradiction between it and effective governance. Decentralization mechanism is an important way proposed by scholars to alleviate the contradiction between the centralized system and effective governance [23]. Since the reform and opening up, the central government has delegated greater power to provincial governments, and the financial relationship between them has been straightened out. With the implementation of decentralization, decentralization among local governments is increasing. However, among provincial, municipal, county, and township governments, financial power is excessively concentrated upward and administrative power is excessively concentrated downward, which hinders the improvement of local government governance performance. In addition to the vertical government hierarchy, the horizontal departmental setup within the government also involves the issue of decentralization. The degree of power concentration and distribution affects the effectiveness of organizational control. When the power of an organization or department is highly concentrated, decisions are made by senior managers, and it is difficult for managers to make accurate decisions due to the limited amount of information. If the power of organizations or departments is decentralized, more grass-roots organizations or people can participate in the decision-making process, which can help reduce the uncertainty of information and make more satisfactory decisions [24]. For example, when several enterprises compete for funds for a government project, the grass-roots government departments or staff often have various business contacts with the enterprise, so they will better understand the real conditions of the enterprise. Therefore, increasing the decision-making power of the grass-roots government departments or staff, such as preliminary review, may reduce the probability of improper allocation of project resources, not only maintaining the reputation of the government departments but also saving the time cost of the enterprise. In addition, enterprises often have some practical difficulties that need to be solved urgently, such as slow-moving products and brain drain, but these difficulties are not within the scope of the work responsibilities of the middle- and high-level government agencies, and the grass-roots government organizations or grass-roots staff lack the actual power to solve problems. Once the grass-roots government is given more powers, the efficiency of enterprises' access to resources may be greatly improved. Based on the above discussion, the following assumptions are put forward:

  H7: the decentralization of government agencies has a positive influence on promoting the acquisition of enterprise policy resources.
  H8: the decentralization of government agencies has a positive influence on promoting the acquisition of financial resources of enterprises.
  H9: the decentralization of government agencies plays a positive influence on promoting enterprises' access to market resources.

The article "Government Structure, Political Connection, and Enterprise Resource Acquisition of Multidimensional Environmental Impact: An Empirical Study Based on the Structural Equation Model" was published in 2022. Journal: J Environ Public Health.

### 3.4. Moderating Role of Political Connection

The relationship system formed by groups or individuals is included in the norms, levels, departments, coordination, power, and other elements of government organizational structure. Enterprise's political connection is one of the important components, which mainly refers to the establishment of good contacts and relationships between enterprises and the government so that enterprises can be protected by the government and reduce the uncertainty in their operations [25, 26]. Specifically, high-level political ties enable enterprises to avoid the predatory behavior of government grass-roots personnel and improve their relative bargaining power when dealing with government officials [27]. If the liaison mechanism between government departments is not smooth, enterprises can offset this negative impact by directly or indirectly establishing contact with government agencies that have control over government departments [28]. For example, when an enterprise applies for a certain qualification standard certification, the grass-roots personnel of the government refuses the application of the enterprise on the ground that there is no relevant certification standard in the region. If the enterprise has a familiar high-level political relationship, it can avoid grass-roots personnel and communicate directly with high-level officials. May be, it can be solved by learning from the certification standards of other regions and adopting the filing system. Even if the business is finally handled by the grass-roots personnel, with the contact of senior officials, the enterprise will increase the probability of successfully handling the business. However, some studies have also shown that the value created by political connections may be weakened by the checks and balances between government departments [5], or political capital may become a negative lift after a sudden change in political structure [29]. Based on the above discussion, the following assumptions are put forward:

  H10: political connection has a positive moderating effect between government structure and enterprise policy resources and market resources. There is a moderating effect between government structure and enterprise financial resources, but there are differences between different dimensions of government structure.

The article "Government Structure, Political Connection, and Enterprise Resource Acquisition of Multidimensional Environmental Impact: An Empirical Study Based on the Structural Equation Model" was published in 2022. Journal: J Environ Public Health.

## 4. Research Design

### 4.1. Data Sources

The data used in this study comes from a questionnaire survey, and the samples were collected from 129 enterprises in F, H, and B cities in A province, S city in H province, and H cities in S province in central China. Among the 129 enterprises, 36 are planting and breeding enterprises, 34 are food trade enterprises, 31 are electronics and technology enterprises, and 28 are machinery manufacturing enterprises. There are 7 enterprises that have been established for more than 15 years, 76 enterprises that have been established for 6 to 15 years, and 46 enterprises that have been newly established for 3 to 5 years. Among them, about 79% are private enterprises, and 94.57% are small- and medium-sized enterprises with less than 200 employees.

There are two reasons for choosing the central region: first of all, the acquisition of external resources of enterprises in the central region can better represent the actual level of China; secondly, the model and operational efficiency of the government structure of neighboring provinces in the central region are similar.

In order to test the appropriateness of the contents of the questionnaire, a pilot test was conducted to determine that these questions are applicable to the political and business environment in central China. The results of the pilot questionnaire show that the respondents are indifferent and the response rate is low. To maximize the reliability of data. First of all, we seek the support of the local Federation of Industry and Commerce, which will provide the list of enterprises under investigation and contact the person in charge of the enterprises; secondly, all selected enterprises have been established for at least 3 years, which is used to reduce the biased answer based on on-off positive or negative experiences [30]. Finally, the interviewees are the senior managers of each enterprise, who know well about the operation of government agencies and enterprises. The time span of this survey is from April 2020 to May 2021, and a total of 387 questionnaires were distributed (among them, there are 141 in the F city, 54 in the H city, 111 in the B city, 39 in the S city, and 42 in the H city). 320 questionnaires were collected, 13 invalid questionnaires were excluded, and finally, 307 valid questionnaires were obtained, with an effective recovery rate of 79%. The 307 respondents were heads or senior managers of 129 enterprises, of which about 67% had college degree or above and the rest had high school or technical secondary school degree. Most of the respondents have worked in this enterprise for at least three years, and only about 14% of the respondents have worked in this enterprise for one year, but have worked in other enterprises. The sample information is shown in Table 1.

The article "Government Structure, Political Connection, and Enterprise Resource Acquisition of Multidimensional Environmental Impact: An Empirical Study Based on the Structural Equation Model" was published in 2022. Journal: J Environ Public Health.

### 4.2. Model Construction and Introduction

#### 4.2.1. Variable Explanation

Based on the domestic and foreign mature scales, according to the interviews with some enterprise executives and heads of government agencies, combined with the organizational chart of government websites, relevant policies, procedures, and related resource allocation publicity information, the variable measurement of this study was evaluated by peer experts, and the measurement scales were determined, all of which were measured by the Likert 5-point method.

*(1) The Explained Variable*. The measurement of this variable divides enterprise resources into three dimensions: policy resources, financial resources, and market resources, and each dimension contains two measurement indicators, which are measured separately.

*(2) Core Variables*. The measurement of this variable takes the government structure as a comprehensive variable composed of three dimensions: formalization, liaison mechanism, and decentralization, and each dimension contains four measurement indicators. Among them, the measurement items of formalization dimension include the government has a clear workflow, the government staff is highly specialized, the government has clear written documents such as policies and systems related to enterprise business, and the government has clear job evaluation standards. The measurement items of the liaison mechanism include the following: the government has formal communication or feedback channels, the government has special liaison departments or personnel for specific projects of enterprises, the government lead agency is responsible for coordinating cross-business of enterprises, and the government specialized agency is responsible for resolving business conflicts of enterprises. The measurement items of decentralization include the following: there are few reporting and approval links for enterprises to handle business, the grass-roots government departments have decision-making power over enterprises' business, the grass-roots government staff have decision-making power over enterprises' business, and the grass-roots government departments can effectively supervise enterprises.

*(3) Adjusting Variables*. This variable is a measure to determine the political connection through the item “in the past three years, the senior executives of affiliated enterprises have established close ties with government officials.”

The article "Government Structure, Political Connection, and Enterprise Resource Acquisition of Multidimensional Environmental Impact: An Empirical Study Based on the Structural Equation Model" was published in 2022. Journal: J Environ Public Health.

#### 4.2.2. Latent Variable and Structural Equation Model

The structural equation model is constructed with formalization (Form), liaison mechanism (Lia), decentralization (Decent), policy resources (Policy), financial resources (Finance), and market resources (Market) as 6 latent variables (see Figure 1). Form, Lia, and Decent each contains four measurement variables, and Policy, Finance and Market each contains two observation variables (see Table 2). *e* represents the residual term.

## 5. Empirical Analysis

### 5.1. Construct Reliability Test

Construct reliability (CR) and average variance extracted (AVE) are called convergence validity, and CR means that the test indicators measuring the same potential trait (construct) will fall on a common factor. Generally speaking, if CR is greater than 0.6 and AVE is greater than 0.5, the questionnaire has good aggregation reliability. Results are shown in Table 3. CR and AVE of all dimensions are basically within the acceptable range, which indicates that the questionnaire has good aggregation reliability.

### 5.2. Structural Validity Test

As for the test results of structural validity, as shown in Table 4, all indicators are within the acceptable range, which is not far from the reference value, indicating that the structural validity of the questionnaire is good.

### 5.3. Discriminant Validity Test

Discriminant validity is a distinguishing index that characterizes each dimension. If there is a significant correlation among the latent variables in the structural equation model and the AVE value under the root sign of each latent variable is greater than the correlation coefficient between each latent variable and other latent variables, it is considered that the questionnaire has good discrimination validity. Results are shown in Table 5. The AVE values under the root signs of the three latent variables are all larger than the correlation coefficient values between themselves and other latent variables, which proves that the discrimination validity of the questionnaire is good.

The article "Government Structure, Political Connection, and Enterprise Resource Acquisition of Multidimensional Environmental Impact: An Empirical Study Based on the Structural Equation Model" was published in 2022. Journal: J Environ Public Health.

### 5.4. Hypothesis Test

#### 5.4.1. The Main Effect

The path coefficients between the core variables and the explained variables are shown in Table 6, and the relationships reflected by them can be summarized as follows: ① the degree of formalization of government structure has a positive effect on enterprises' access to policy resources. Hypothesis 1 is supported. Although the positive effect of formalized structure on financial resources is weakly significant, the conclusion of hypothesis 2 can also be confirmed. However, the impact of standardized structure on enterprise market resources is not significant. Therefore, hypothesis 3 is not supported. ② The effect of liaison mechanism on enterprise policy resources is not significant, and hypothesis 4 is not supported. The liaison mechanism is conducive to the acquisition of financial resources, and hypothesis 5 is proved. The impact of liaison mechanism on enterprise market resources is positively and weakly significant, and hypothesis 6 is supported. However, the impact on enterprise policy resources is not significant. Therefore, hypotheses 5 and 6 are confirmed. ③ Decentralization has a significant positive impact on the acquisition of enterprise policy resources and market resources, but not on enterprise financial resources. Therefore, assumptions 7 and 9 are true, but assumption 8 is not.

#### 5.4.2. Regulation

The adjustment variable “political connection” is multiplied by four questions in each dimension of the independent variable, and the adjustment interaction item is constructed. And, verify the significance of the path coefficients of the moderators to policy resources, financial resources, and market resources. The model (see Figure 2) and path coefficients (see Table 7) are as follows. Table 7 shows that political ties play a positive role in regulating the various dimensions of government structure, enterprise policy resources, and market resources, while the interaction between formalization and liaison mechanism and political ties has no significant impact on enterprise financial resources. But the interaction between decentralization and political ties has a significant positive impact on enterprise financial resources. Therefore, hypothesis 10 is supported.

## 6. Conclusion and Enlightenment

How does the government structure affect the acquisition of enterprise resources? Through the analysis of 307 observations of 129 enterprises in central China, this paper finds that the formalized structure has a significant positive impact on the acquisition of enterprise policy resources, the liaison mechanism has a significant positive impact on the acquisition of enterprise financial resources, and the decentralization of power has a significant positive impact on the acquisition of enterprise policy resources and market resources. The formalized structure has a weak significant positive impact on the acquisition of financial resources, and the liaison mechanism has a weak significant positive impact on the acquisition of market resources. At the same time, political connection can amplify the positive effects of the three structural elements on enterprise resource acquisition, and even for variables that had no connection, such as formalization structure and enterprise market resources, decentralization, and enterprise financial resources, political connection has played a significant positive role in regulating.

The article "Government Structure, Political Connection, and Enterprise Resource Acquisition of Multidimensional Environmental Impact: An Empirical Study Based on the Structural Equation Model" was published in 2022. Journal: J Environ Public Health.

The core contribution of this paper is reflected in three aspects. Firstly, this paper provides a new idea for the study of multidimensional political factors affecting enterprise resource acquisition. The existing literature fails to consider the influence of government structure on enterprise resource acquisition and ignores the uncontrollable factors in enterprise resource acquisition. At the same time, due to the abstraction and complexity of the concept of organizational structure itself, academic circles rarely use quantitative methods to study organizational structure. Based on the three elements of government structure, such as formalization, liaison mechanism, and decentralization, this paper empirically analyzes their relationship with the political resources of enterprises and their influence degree.

Secondly, the paper points out the influence of the correct operation mode of government structure on enterprise development. When the government structure runs in a reasonable and efficient way, that is, its dimensions such as formalization, liaison mechanism, and decentralization are in a good state, both enterprises and the government benefit. For example, when a government agency conducts public service bidding, the formalization process brings reasonable and fair enterprise competition, and the government can complete the project construction at the lowest cost. Also, enterprises can put more resources into the improvement of market capacity and achieve long-term development.

Finally, the article provides a way to solve the structural obstacles of government institutions. During the period of China's transition, weak administrative institutions have created some structural obstacles. For example, the irregularities of government behavior still exist. The checks and balances between government departments weaken their ability to provide resources for enterprises; Slow public sector system may lead to the delay of approval. When power is highly concentrated, enterprises may be exploited from the grass-roots level and so on. Therefore, this kind of environment makes it necessary for enterprises to establish appropriate political ties. Through the political connection of enterprises, the uncertainty caused by structural obstacles can be reduced, and opportunities for obtaining resources can be created. However, enterprises cannot rely too much on the political ties established with the government in terms of resource acquisition. Excessive political ties will lead to increased operating costs and bribery and corruption, or inappropriate political connection leads to excessive power of enterprises, such as excessive use of public resources to enhance competitive advantage and excessive discretion of enterprise executives.

The article "Government Structure, Political Connection, and Enterprise Resource Acquisition of Multidimensional Environmental Impact: An Empirical Study Based on the Structural Equation Model" was published in 2022. Journal: J Environ Public Health.

The findings of this paper have important management implications for the reform of government structure and how to build the relationship between enterprises and the government. First of all, the government structure needs to continue to deepen the reform in the following three aspects: (1) scientific, procedural, and transparent government normative acts based on legal basis. (2) Cooperation and linkage between government departments. (3) Decentralization based on unified leadership. Secondly, in order to prevent the negative impact of government structural obstacles on enterprise resource acquisition, enterprises must have certain political ability, that is, regardless of the state of government structure; enterprises can identify different types of political problems and take different actions. There are two main ways to develop and cultivate the political ability of enterprises. (1) Previous experience: enterprises can learn to make better use of political strategies by summing up their experiences in dealing with government agencies [31]. (2) Market ability: on the basis of market ability, enterprises develop directly related political ability, which can reduce the cost of political contact. Of course, under the environment of perfect government structure elements, the market ability of enterprises can replace the function of their political ability, so as to realize the acquisition of enterprise resources.

Due to the limitation of conditions, there are still some research limitations in this paper, which need further research in the future. (1) The area where the sample is located can be further expanded. In the future, small- and medium-sized enterprises and government agencies in the east and south can be included in the research scope, and a more meaningful conclusion may be obtained by comparative analysis with the situation in the central and western regions. (2) Combining the case analysis with the questionnaire survey can not only ensure the universality of the conclusion but also help to create a new theory, which is more effective.

The article "Government Structure, Political Connection, and Enterprise Resource Acquisition of Multidimensional Environmental Impact: An Empirical Study Based on the Structural Equation Model" was published in 2022. Journal: J Environ Public Health.

## Figures and Tables

**Figure 1:** SEM model (established by AMOS).

**Figure 2:** SEM model (including adjustment variables).

**Table 1:** Basic information of samples.

Index	Basic feature	Times	Ratio (%)
Enterprise nature	State-owned enterprise	16	112.4
	Full foreign-owned enterprises	11	8.5
	Private enterprise	102	79.1

Enterprise establishment time	3–5 years	446	35.7
	6–9 years	557	44.2
	10–15 years	119	14.7
	More than 15 years	7	5.4

Education level of interviewees	High school or technical secondary school	101	32.9
	Universities and colleges	135	44
	Undergraduate course	54	17.6
	Masters	17	5.5

Enterprise scale	≤20 people	28	21.7
	21–50 people	59	45.74
	51–100 people	27	20.93
	101–200 people	8	6.2
	201–500 people	4	3.1
	More than 500 people	3	2.33

Industry nature	Planting and breeding	36	27.9
	Food and commerce	34	26.4
	Electron	16	12.4
	Science and technology	15	11.6
	Machinery manufacturing	28	21.7

**Table 2:** Latent variables and observed variables.

Latent variable	Observation variable	Coding
Formalization	Workflow	G1
	Professionalization	G2
	Policies and systems	G3
	Evaluation criterion	G4

Liaison mechanism	Communication channel	X1
	Specific contact	X2
	Work crossing	X3
	Work conflict	X4

Decentralization	Approval link	Q1
	Grass-roots department	Q2
	Grass-roots personnel	Q3
	Grass-roots supervision	Q4

Policy resources	Policy information	Z1
	Government subsidy	Z2

Financial resources	External financing	C1
	Interest-free loan	C2

Market resources	Market expansion	S1
	Talent acquisition	S2

**Table 3:** Construct reliability.

Path			Path coefficient	CR	AVE
Workflow	<---	Form	0.809	0.942	0.803
Professionalization	<---	Form	0.965		
Policies and systems	<---	Form	0.917		
Evaluation criterion	<---	Form	0.886		

Communication channels	<---	Lia	0.897	0.942	0.803
Specific contact	<---	Lia	0.992		
Work crossing	<---	Lia	0.841		
Work conflict	<---	Lia	0.847		

Approval link	<---	Decent	0.871	0.947	0.817
Grass-roots department	<---	Decent	0.886		
Grass-roots personnel	<---	Decent	0.966		
Grass-roots supervision	<---	Decent	0.890		

Policy Information	<---	Policy	0.755	0.705	0.545
Government subsidy	<---	Policy	0.721		

External Financing	<---	Finance	0.580	0.616	0.449
Interest-free loan	<---	Finance	0.749		

Market expanding	<---	Market	0.588	0.701	0.549
Talent acquisition	<---	Market	0.867		

The article "Government Structure, Political Connection, and Enterprise Resource Acquisition of Multidimensional Environmental Impact: An Empirical Study Based on the Structural Equation Model" was published in 2022. Journal: J Environ Public Health.

**Table 4:** Structural validity.

Model fit		Recommended values	Measurement model
Absolute fit	GFI	>0.9	0.827
	AGFI	>0.9	0.759
	RMSEA	<0.08	0.107

Baseline comparisons	NFI	>0.9	0.887
	RFI	>0.9	0.860
	IFI	>0.9	0.910
	TLI	>0.9	0.888
	CFI	>0.9	0.910

Parsimony-adjusted measures	PGFI	>0.5	0.595
	PNFI	>0.5	0.713
	CMIN/DF	<5	4.503

**Table 5:** Discriminant validity.

	Form	Lia	Decent	Policy	Finance	Market
Form	0.803					
Lia	0.436	0.803				
Decent	0.564	0.708	0.817			
Policy	0.409	0.227	0.383	0.545		
Finance	0.267	0.329	0.264	0.051	0.449	
Market	0.239	0.393	0.383	0.074	0.127	0.549
SQRT (AVE)	0.896	0.896	0.904	0.738	0.670	0.741

**Table 6:** Estimation results of path and load coefficient.

Path			Estimate	SE	CR	*P*	Label
Policy	<---	Form	0.158	0.038	4.175	<0.001	Sig
Finance	<---	Form	0.058	0.027	2.16	0.031	Weak sig
Market	<---	Form	−0.009	0.026	−0.331	0.741	No sig
Policy	<---	Lia	−0.058	0.036	−1.597	0.11	No sig
Finance	<---	Lia	0.1	0.029	3.404	<0.001	Sig
Market	<---	Lia	0.057	0.027	2.078	0.038	Weak sig
Policy	<---	Decent	0.142	0.041	3.472	<0.001	Sig
Finance	<---	Decent	−0.004	0.028	−0.141	0.888	No sig
Market	<---	Decent	0.109	0.033	3.313	<0.001	Sig

**Table 7:** Adjustment variable path coefficient table.

Path			Estimate	SE	CR	*P*	Label
Policy	<---	Form moderator	0.081	0.013	6.184	<0.001	Sig
Finance	<---	Form moderator	0.016	0.01	1.671	0.095	No sig
Market	<---	Form moderator	0.032	0.01	3.18	0.001	Sig
Policy	<---	Lia moderator	0.042	0.009	4.522	<0.001	Sig
Finance	<---	Lia moderator	0.004	0.007	0.625	0.532	No sig
Market	<---	Lia moderator	0.038	0.008	4.783	<0.001	Sig
Policy	<---	Decent moderator	0.042	0.018	2.383	0.017	Sig
Finance	<---	Decent moderator	0.053	0.015	3.528	<0.001	Sig
Market	<---	Decent moderator	0.025	0.012	2.033	0.042	Sig

## Data Availability

All data used to support the findings of the study are included within this article.
